RETRACTED

# Osteogenic protein-1 attenuates apoptosis and enhances matrix synthesis of nucleus pulposus cells under high magnitude compression though inhibiting the p38 MAPK pathway

**DOI:** 10.1042/BSR20180018

**Published:** 2018-03-16

**Authors:** Haolin Fang, Xianzhou Li, Haiming Shen, Buwei Sun, Haijun Teng, Pei Li

**Affiliations:** 1 Department of Emergency Trauma Surgery, Jining No.1 People’s Hospital, Jining 272011, P.R. China; 2 Department of Spinal Surgery, Jining No.1 People’s Hospital, Jining 272011, P.R. China; 3 Department of Neurosurgery, Jining No.2 People’s Hospital, Jining 272011, P.R. China; 4 Department of Orthopaedics, Jining No.2 People’s Hospital, Jining 272011, P.R. China; 5 Department of Orthopaedics, No.89 Hospital of PLA, Weifang, Shandong 261026, P.R. China

**Keywords:** apoptosis, compression, matrix, nucleus pulposus, osteogenic protein-1

## Abstract

Disc degeneration is correlated with mechanical load. Osteogenic protein-1 (OP-1) is potential to regenerate degenerative disc. To investigate whether OP-1 can protect against high magitude compression-induced nucleus pulposus (NP) cell apoptosis and NP matrix catabolism, and its potential mechanism; porcine discs were cultured in a bioreactor and compressed at a relatively high-magnitude mechanical compression (1.3 MPa at a frequency of 1.0 Hz for 2 h once per day) for 7 days. OP-1 was added along with the culture medium to investigate the protective effects of OP-1. NP cell apoptosis and matrix biosynthesis were evaluated. Additionally, activity of the p38 MAPK pathway is also analyzed. Compared with the control group, high magnitude compression significantly promoted NP cell apoptosis and decreased NP matrix biosynthesis, reflected by the increase in the number of terminal deoxynucleotidyl transferase dUTP nick-end labeling (TUNEL)-positive cells and caspase-3 activity, the up-regulated expression of *Bax* and *caspase-3* mRNA and down-regulated expression of *Bcl-*2 mRNA, and the decreased Alcian Blue staining intensity and expression of matrix proteins (aggrecan and collagen II). However, OP-1 addition partly attenuated the effects of high magnitude compression on NP cell apoptosis and NP matrix biosynthesis. Further analysis showed that inhibition of the p38 MAPK pathway partly participated in this process. OP-1 can attenuate high magnitude compression-induced NP cell apoptosis and promoted NP matrix biosynthesis, and inhibition of the p38 MAPK pathway may participate in this regulatory process. The present study provides that OP-1 may be efficient in retarding mechanical overloading-exacerbated disc degeneration.

## Introduction

Intervertebral disc degeneration (IDD) is a worldwide disease that leads to numerous socioeconomic loss and a heavy burden on the healthcare system [1]. It is regarded as a main cause of low back and leg pain, which interferes with normal daily activities and significantly impacts the ability (of patients) to work [2]. Recently, many basic research teams are devoting their efforts to biologically regenerate the degenerative disc and retard the speed of disc degeneration.

RETRACTED

The intervertebral disc functions as a connection structure between two adjacent vertebral bones and it plays an important role in transmitting and absorbing the mechanical load [3]. Previous studies have demonstrated that the disc nucleus pulposus (NP) region first exhibits degenerative changes during the disc degeneration process, amongst which cellular apoptosis and matrix biosynthesis decline are two common pathological features of the degenerative disc NP tissue [4,5]. Because the NP matrix is mainly produced by the NP cells with normal biological activity, many scholars deduce that inhibition of NP cell apoptosis and activation of matrix biosynthesis potency may be effective to maintain the normal disc function.

According to previous studies, mechanical overload is the most common risk factor of disc degeneration [6,7]. A previous study showed that a high magnitude compression can increase NP cell apoptosis and decreased NP matrix synthesis in a disc organ culture system [8]. Additionally, the p38 MAPK pathway is reported to be involved in the mechanical load-induced disc degenerative changes [9,10]. Several growth factors including insulin-like growth factor-1 (IGF-1), basic fibroblast growth factor (bFGF), and transforming growth factor-β (TGF-β) have shown protective effects on cell viability and matrix anabolism [11–13]. Osteogenic protein-1 (OP-1), also named as bone morphogenetic protein-1, is a member of TGF-β superfamily. Recent *in vitro* and *in vivo* studies have demonstrated that OP-1 is helpful to stimulate matrix production of NP cells and retarding disc degeneration in animal models [14,15]. In the present study, we mainly aimed to investigate whether OP-1 can attenuate NP cell apoptosis and promote NP matrix synthesis under the high-magnitude compression in a previously described disc organ culture and the potential mechanism behind this process.

## Materials and methods

### Ethical statement

All experimental animals were used according to the guidelines of the Ethics Committee at Jining No. 2 People’s Hospital (SWFK (LU) 2062-0016).

### Disc harvest and organ culture

The intact discs (Th11/Th12-L4/L5) were isolated from 15 healthy pigs (male, 10–13 kg, 3–4 months old) according to a previous study [16]. After the discs were separated, the attached ligament and connective tissue were further removed under a dissecting microscope. Thereafter, the isolated discs were perfusion-cultured for 7 days in the culture chambers of a perfusion and mechanically active bioreactor [17]. In the meantime, the discs were compressed at a relatively high magnitude of 1.3 MPa at a frequency of 1.0 Hz for 2 h once per day. Because 1.3 MPa of compressive magnitude was reported to significantly promote NP cell apoptosis and matrix catabolism, it was used as a high magnitude of mechanical compression in this study [16]. In addition, to investigate the effects of OP-1 on NP cell apoptosis and matrix synthesis under this high magnitude compression, the compressed discs were incubated with OP-1 (100 ng/ml) that was designed according to the previous studies [18,19]. The unloaded discs were regarded as the controls. Fresh DMEM/F12 culture medium (Gibco, U.S.A.) supplemented with 10% (v/v) FBS (Gibco, U.S.A.) and 1% (v/v) penicillin-streptomycin (Gibco, U.S.A.) was circulated at a rate of 5 ml/min. Importantly, because the disc samples was limited due to the limited experimental animals, discs from the same levels were used for the same assay as described previously to avoid the interference between different vertebral levels [20]. For example, the biochemical content measurement assay was performed on the same three discs (L2/3, L3/4, and L4/5) from different animals.

RETRACTED

### Terminal deoxynucleotidyl transferase dUTP nick-end labeling assay

Briefly, discs were fixed with 4% paraformaldehyde, decalcified with 10% EDTA, and embedded in paraffin. After disc cross-sections were prepared, they were permeated with proteinase K. Then, terminal deoxynucleotidyl transferase dUTP nick-end labeling (TUNEL) staining assay was performed according to the manufacturer’s instructions (Roche, Switzerland). Staining-positive NP cells were observed under a light microscope and quantitated with the ImagePro Plus software (version 5.1, Media Cybernetics, Inc.).

### Caspase-3 activity measurement

Briefly, the central gelatinous NP samples were isolated after disc organ culture and incubated with 300 μl lysis buffer for 10 min. Then, the protein supernatant was separated by centrifugation at 15000 ***g*** for 15 min at 4°C. Thereafter, the reaction system containing 40 μl buffer, 50 μl lysate, and 10 μl Ac-LEHD-*p*NA was incubated for 8 h at 37°C. Finally, caspase-3 activity was calculated by measuring the absorbance value at a wavelength of 405 nm.

### Alcian Blue staining assay

Briefly, previously prepared disc cross-sections were first dewaxed with xylene and rinsed with PBS. Then, Alcian Blue assay was performed according to the manufacturer’s instructions. All the disc sections were observed under a light microscope and the staining intensity was quantitated using the ImagePro Plus software (version 5.1, Media Cybernetics, Inc.).

RETRACTED

### Biochemical content measurement

After disc organ culture, the central NP tissue was isolated as described above to measure the glycosaminoglycan (GAG) and hydroxyproline (HYP) contents. Briefly, one part of NP samples was lyophilized for 24 h, and digested at 60°C for 24 h in 1 ml water containing 5 mg/ml papain, 0.2 mol/l NaCl, 0.01 mol/l cysteine hydrochloride, 0.1 mol/l CH_3_COONa, and 0.05 mol/l Na_2_-EDTA (Sangon, Biotech Co., Ltd., China). Then, the GAG content was calculated using a dimethyl methylene blue (DMMB) assay [21]. Another part of NP samples was weighed to determine their wet weights, and then the HYP content was determined using an HYP quantitation kit (Nanjing Jiancheng, China) according to the manufacturer’s instructions.

### Real-time PCR analysis

Briefly, total RNA was extracted from the isolated NP tissue using the TRIzol reagent (Invitrogen, U.S.A.) and synthesized into cDNA using the PrimeScript™ II First Strand cDNA Synthesis Kit (Takara, Japan). Then, the PCR was performed on a reaction mixture (20 μl) containing 10 μl SYBR Green Mix (TOYOBO, Japan), 8 μl RNase-free water, 1.5 μl cDNA, and 1 μl primer mix. The reaction parameters were: 3 min at 95°C, followed by 35 amplification cycles of 15 s at 95°C, 10 s at 56°C, and 15 s at 72°C. Gene-specific primers (Table 1) were designed and synthesized by a domestic commercial company (Sangon, Biotech Co., Ltd., China). GAPDH was used as an internal control. The relative expression of target genes was expressed according to the method 2^―ΔΔ*C*^_t_.

**Table 1:** Primers of target genes

Gene	Accession number	Forward (5′–3′)	Reverse (5′–3′)
*GAPDH*	NM_001082253.1	GACCACTTTGTGAAGCTCATTTC	GTGGTTTGAGGGCTCTTACTC
*Bcl-2*	XM_003121700.3	GGGAGGATTGTGGCCTTCTT	GGCCCATACAGCTCCACAAA
*Bax*	XM_003355975.2	TTCATCCAGGATCGAGCAGG	TCCAATGCGCTTGAGACACT
*Caspase-3*	NM_214131.1	GGGATTGAGACGGACAGTGG	TGAACCAGGATCCGTCCTTTG
*Aggrecan*	NM_001164652.1	CGTGGTCCAGCACTTCTAAA	AGTCCACTGAGATCCTCTACAC
*Collagen II*	XM_001925959.4	CCGGGTGAACGTGGAGAGACTG	CGCCCCCACAGTGCCCTC

### Western blotting assay

Briefly, total protein was extracted using the RIPA lysis buffer (Beyotime, China) and subjected to the SDS/PAGE system (6% separate gel). After the protein sample was transferred on to the PVDF membranes, the PVDF membranes were sequentially incubated with primary antibodies (GAPDH: Abcam, ab8245; collagen II: Abcam, ab34712; aggrecan: Santa Cruz Biotechnology, sc-16492; SOX9: Abcam, ab185966. All primary antibodies were diluted at 1:1000) at 4°C overnight, and the corresponding HRP-conjugated secondary antibodies (goat anti-mouse IgG, goat anti-rabbit IgG, and mouse anti-goat IgG, ZSGB-BIO, China, diluted at 1:1000) at room temperature for 2 h. Finally, ECL Plus reagent (Thermo, U.S.A.) was used to develop the protein bands on PVDF membranes. After the gray value of protein bands was calculated using the ImageJ software (National Institutes of Health, U.S.A.), it was normalized to that of GAPDH.

RETRACTED

### Statistical analysis

Each test in the present study was performed at least three times to ensure repeatability. All data expressed as mean ± S.E.M. were analyzed using SPSS 17.0 software. After the homogeneity test for variance, intergroup difference was analyzed by the one-way ANOVA and the post hoc test was performed using the LSD test. A difference was considered statistically significant if the *P*-value<0.05.

## Results

### TUNEL assay

TUNEL positive-stained NP cells were regarded as the apoptotic NP cells. Results showed that the number of apoptotic NP cells in the compression group was increased compared with the control group. However, the addition of OP-1 obviously decreased the number of apoptotic NP cells in the compression group (Figure 1).

**Figure 1:** NP cell apoptosis evaluated by TUNEL staining assay Magnification: 200×; scale = 100 μM; *n*=3. Data are expressed as mean ± S.D. *, Indicates a significant difference (*P*<0.05) between two groups.

### Caspase-3 activity

The caspase-3 is one of the pivotal enzymes in the cell apoptosis process [22]. Our results showed that caspase-3 activity was significantly increased in the compression group, but partly decreased by the addition of OP-1 under this high magnitude compression (Figure 2).

**Figure 2:** Caspase-3 activity measurement Data are expressed as mean ± S.D. *, Indicates a significant difference (*P*<0.05) between two groups.

### Alcian Blue staining

Alcian Blue staining is a common method to indicate the production and distribution of proteoglycan in cartilaginous tissue [23]. In this study, this high magnitude compression significantly decreased the staining intensity of the Alcian Blue. However, OP-1 partly increased the staining intensity of Alcian Blue under this high magnitude compression (Figure 3).

**Figure 3:** Proteoglycan content observation by Alcian Blue staining assay Magnification: 200×; scale = 100 μM; *n*=3. Data are expressed as mean ± S.D. *, Indicates a significant difference (*P*<0.05) between two groups.

### GAG and HYP content

GAG and HYP are common biochemical compositions within the disc NP region. Results showed that both GAG content and HYP content in the compression group were decreased under this high magnitude compression. However, they were increased by the addition of OP-1 in the compression group (Figure 4).

RETRACTED

**Figure 4:** Biochemical content measurement Data are expressed as mean ± S.D., *n*=3. *, Indicates a significant difference (*P*<0.05) between two groups.

### Gene expression

According to the previous opinion, aggrecan and collagen II are main matrix proteins within the disc NP tissue [24]. In this study, gene expression of aggrecan, collagen II, and SOX-9 are down-regulated by this high magnitude compression. However, OP-1 significantly up-regulated their expression under this high magnitude compression (Figure 5).

**Figure 5:** Real-time PCR analysis Gene expression of NP matrix molecules (aggrecan and collagen II) and apoptosis-related molecules (Bcl-2, Bax, and caspase-3). Data are expressed as mean ± S.D., *n*=3. *, Indicates a significant difference (*P*<0.05) between the two groups.

### Western blotting assay

Results showed that protein expression of both aggrecan and collagen II were decreased in the compression group, whereas they were up-regulated by the addition of OP-1 in the compression group (Figure 6). Additionally, we found that this high magnitude compression significantly decreased activity of the p38 MAPK pathway, whereas the addition of OP-1 partly increased activity of the p38 MAPK pathway under mechanical compression (Figure 7).

**Figure 6:** Protein expression of NP matrix molecules (aggrecan and collagen II) Data are expressed as mean ± S.D., *n*=3. *, Indicates a significant difference (*P*<0.05) between two groups.

**Figure 7:** Activation of the p38 MAPK pathway amongst the groups Data are expressed as mean ± S.D., *n*=3. *, Indicates a significant difference (*P*<0.05) between two groups.

## Discussion

In the present study, we investigated the positive effects of OP-1 against high magnitude compression-induced NP cell apoptosis and NP matrix decline. To our knowledge, few studies focussed on the biological effects of OP-1 on disc NP cell activities under the mechanical compression. Our results confirmed the previous study that high magnitude compression promotes NP cell apoptosis and inhibits NP matrix synthesis. Additionally, we also found that OP-1 could alleviate the unfavorable effects of high magnitude compression on NP cell viability and matrix biosynthesis in a disc organ culture. The present study provides clues that OP-1 may be a potential drug to alleviate mechanical overloading-induced disc NP tissue degeneration.

Dynamic compression is one form of the main mechanical conditions experienced by the discs *in vivo* [25]. During the past years, many scholars have measured the intradisc pressure under the different body postures and these crude data have indicated that one body posture which causes a high intradisc pressure may trend to induce and/or accelerate disc degeneration [26–29]. Additionally, lot of researchers have performed some basic studies and reported that mechanical overloading is one of important external risk factor of disc degeneration [30]. In this study, 1.3 MPa of compression magnitude is also within the range of physical intradisc pressure and has been reported to do harms to NP cell viability and NP matrix biosynthesis [8]. Because the NP region first exhibits degenerative changes during disc degeneration [4,5], we mainly focussed on the NP tissue even though the intact disc consists of the three structurally integrated parts, such as NP tissue, annulus fibrosus tissue, and cartilage endplates.

RETRACTED

Current treatments for disc degeneration are mainly aimed to alleviate pain symptom but not to re-establish the biological functions of the disc. Growth factor is potential to increase disc cell viability and promote matrix biosynthesis. In a previous systematic review, OP-1 is reported to be effective in retarding disc degeneration and regenerating discs [14]. However, whether it can protect disc NP cells under the condition of mechanical overloading is unknown. In the present study, we found that high magnitude compression significantly increased TUNEL-positive cells and caspase-3 activity, down-regulated gene expression of Bcl-2 and up-regulated gene expression of Bax and caspase-3 in NP cells, whereas OP-1 addition partly attenuated these trends under high magnitude compression. These findings confirm again that mechanical overloading can promote disc cell death and directly suggest that OP-1 may be effective to regenerate mechanical overloading-induced disc NP cell apoptosis. This is, to some extent, similar to a previous study that OP-1 was able to decrease TNF-α and/or H_2_O_2_-induced disc cell apoptosis [15].

Matrix production decrease and degradation increase are also classical features during disc degeneration [4]. Previous studies demonstrated that mechanical overloading significantly decreases matrix synthesis and increases matrix degradation [8]. The decreased matrix biosynthesis activity in the present study is in line with those previous studies. However, we simultaneously found that OP-1 addition was able to increase Alcian Blue staining intensity, matrix protein expression, and gene expression in NP cells under the high magnitude compression, suggesting that OP-1 is promising to inhibit mechanical overloading-induced disc NP matrix degradation. In line with this, a previous study showed that OP-1 injection was able to inhibit disc matrix catabolic metabolism in a compressive loading-induced disc degeneration model [31,32].

RETRACTED

The p38 MAPK signaling pathway belongs to the MAPK signaling pathways that translate extracellular stimulations into intracellular responses, which affects cell viability and cell biosynthesis via alterations in the activity of specific transcription factors [33]. A previous study has showed that high magnitude compression can activate the p38 MAPK pathway to accelerate disc NP cell senescence and thus decrease NP cell matrix biosynthesis in a disc perfusion culture [9]. This study suggests that the activation of p38 MAPK pathway may be responsible for the harmful effects of mechanical overloading on the disc NP cells. In the present study, we also found that activity of the p38 MAPK pathway was significantly increased under the high magnitude compression. However, OP-1 addition obviously decreased activity of the p38 MAPK pathway under the high magnitude compression. Combined with the decreased NP cell apoptosis ratio and increased NP matrix biosynthesis after the OP-1 is added into the culture medium under high magnitude compression, we deduce that OP-1 may attenuate NP cell apoptosis and increase NP matrix biosynthesis through inhibiting the p38 MAPK pathway under high magnitude compression.

The present study also has several limitations. First, lot of notochordal cells are within the pig disc NP tissue. Their existence may affect the response of NP cells to the mechanical compression. Hence, the present results may be a little different from the actual results under mechanical compression. Second, the present study is an *in vitro* study. An additional *in vivo* animal study is needed to verify the present results.

## Conclusion

In conclusion, we demonstrate that OP-1 is able to attenuate NP cell apoptosis and promote NP matrix biosynthesis under the high magnitude compression in the disc bioreactor culture, and the inhibition of the p38 MAPK pathway may be involved in this regulatory process. The present study indirectly provides that OP-1 may be a potential drug to alleviate mechanical overloading-induced disc NP tissue degeneration.

## Abbreviations

DMEM/F12: Dulbecco’s modified Eagle medium/nutrient mixture F-12
GAG: glycosaminoglycan
GAPDH: glyceraldehyde-3-phosphate dehydrogenase
HRP: horseradish peroxidase
HYP: hydroxyproline
NP: nucleus pulposus
OP-1: osteogenic protein-1
TGF-β: transforming growth factor-β
TNF-α: tumor necrosis factor-α
TUNEL: terminal deoxynucleotidyl transferase dUTP nick-end labeling
